RETRACTED

# Effect of High-Quality Nursing Intervention on the Quality of Life and Psychological State of Tumor Patients Undergoing First Chemotherapy

**DOI:** 10.1155/2022/9466665

**Published:** 2022-06-25

**Authors:** Huaqin Ding, Yuanxia Jiang

**Affiliations:** Department of Oncology, Jiangyin Hospital of Traditional Chinese Medicine, Jiangyin, Wuxi, Jiangsu Province, China

## Abstract

This study aimed to investigate the effect of high-quality nursing intervention on the quality of life (QOL) and psychological state of patients undergoing chemotherapy for the first time. A total of 100 malignant tumor patients admitted to Jiangyin Hospital of Traditional Chinese Medicine to receive chemotherapy for the first time from October 2018 to July 2020 were selected and randomized either to the control group or to the study group (50 cases in each group) via the random number table method. The control group received routine nursing, while the study group received high-quality nursing intervention. There was no striking difference in self-rating anxiety scale (SAS), self-rating depression scale (SDS), Karnofsky score (KPS), Eastern Cooperative Oncology Group (ECOG), and QOL between the two groups before nursing intervention (all *P* > 0.05). After nursing intervention, the SAS, SDS, KPS, ECOG, and QOL in the study group were better than those in the control group (all *P* < 0.05). The adverse reaction scores of the patients in the study group were lower than those in the control group (*P* < 0.05). High-quality nursing intervention can effectively reduce the psychological pressure of the first chemotherapy for patients with malignant tumor, ameliorate the psychological burden of patients, relieve patients' anxiety and fear, thus improve the chemotherapy effect, and contribute to improve their QOL.

## 1. Introduction

A malignant tumor is a health concern that imposes considerable threats on human beings [1, 2]. The malignant tumor features infinite proliferation, and it would wildly proliferate if effective measures are not provided. In addition, a malignant tumor is also invasive and metastatic and can invade surrounding organs, such as adjacent blood vessels and organs [3, 4]. Chemotherapy is currently a conventional method for the treatment of malignant tumors. Although chemotherapy can treat malignant tumors clinically, it is associated with certain psychological and physical damage [5]. Therefore, patients receiving first chemotherapy are prone to negative moods such as worry and anxiety, and even depression in severe cases. Such psychological emotions hinder the recovery of the patient and hobble the implementation of treatment. With the rapid development of economy and medical quality, patients and their families are highly demanding on the quality of clinic nursing, and the provision of high-quality nursing services is a key factor to improve patients' physical recovery. Clinical high-quality nursing intervention is a nursing mode of patients centered to strengthen basic nursing, comprehensively implement nursing responsibility system, deepen nursing professional connotation, and improve nursing service level as a whole. As previously reported, clinical high-quality nursing interventions have significant effects on improving patients' psychological emotions, QOL, and treatment effects [6, 7]. The purpose of this study was to investigate the impact of high-quality nursing intervention on the QOL and psychological state of patients undergoing chemotherapy for the first time and to provide reference for clinical practice.

RETRACTED

## 2. Materials and Methods

### 2.1. Baseline Data

A total of 100 malignant tumor patients admitted to our hospital to receive chemotherapy for the first time from October 2018 to July 2020 were selected and randomized either to the control group or to the study group (50 cases in each group). The research was approved by the Ethics Committee of the Jiangyin Hospital of Traditional Chinese Medicine, No. JY2883.

### 2.2. Nursing Methods

The patients in the control group received routine nursing intervention, including informing the patients about the relevant knowledge and precautions of disease and chemotherapy. The changes in patients' physical signs were strictly monitored, and medication and diet were guided.

The patients in the study group adopted high-quality nursing intervention. The detailed nursing contents are as follows. ① Psychological nursing intervention upon admission: the medical staff gave an introduction to patients and their families about the ward environment, basic knowledge of diseases, chemotherapy procedures, the necessity and importance of auxiliary examinations, and the basic information of the attending doctor, to eliminate a sense of unfamiliar to the environment, further build trust and compliance toward nursing staff, improve the adherence with nursing and treatment work, and finally lay a solid foundation for the establishment of a harmonious nurse-patient relationship. Then, the medical staff presented successful cases of treatment to help patients establish confidence to overcome the disease and to receive treatment with a positive mentality. ② Psychological nursing intervention before chemotherapy: the medical staff introduced the effect of chemotherapy and possible discomfort to the patient, to guide the patient in physical relaxation and mental guidance, and encouraged family members to actively participate in psychological intervention, to improve family warmth and support for the patient, reduce the patient's psychological pressure, relieve the patient's negative emotions, and actively cooperate with the treatment. ③ Postchemotherapy psychological nursing intervention: the medical staff gave professional explanations for the adverse reactions of the patients to maintain emotional stability, guide them to learn how to deal with physical discomfort, and firmly believe in the effectiveness of the treatment; according to mobilizing family members to accompany, it could create a relaxed atmosphere, eliminate the patient's sense of guilt dragging down the family, let the patient feel the care of the family, and enhance the patient's confidence in treatment; according to the patient's own situation, professional nursing support and dietary guidance should be given to avoid the intake of spicy and irritating food, to ensure balanced nutrition, enhance physical resistance, and promote recovery [8]. ④ Adverse reaction nursing intervention: (1) phlebitis nursing—after chemotherapy, a small amount of normal saline is used to rinse the tube, and 250 ml of normal saline is used for rapid intravenous infusion, which can dilute the residual chemotherapy drugs on the vascular wall, reduce the stimulation to local tissues, and effectively prevent phlebitis. To reduce the occurrence of phlebitis, it is necessary to adjust the intravenous drip speed and select the vein and deep vein catheterization. (2) Gastrointestinal reaction nursing—patients with loss of appetite should be given a high-protein, high-vitamin, high-calorie diet, such as eggs, lean meat, fresh vegetables, and fruits. If diarrhea symptoms occur, it is necessary to give a refined perianal care, make perianal skin clean and dry, avoid dairy products and high-fat food, eat light, easy-to-digest liquid food, and medication can be given. For those who are afraid of eating due to vomiting, favorable places should be provided so that they can cooperate well with eating. (3) Bone marrow suppression nursing—during chemotherapy, patients are recommended to live in a single room and reduce visits, and nurses pay attention to changes in blood routine, prevent infection, and do basic care, such as keeping oral cavity clean, cutting nails regularly, and changing clothes and gowns frequently. In case of anemia, the patient should be given component blood transfusion, and the patient's temperature should be closely observed. If the WBC is lower than 1.0 × 10^9^, protective isolation measures should be taken to avoid cross-infection.

RETRACTED

### 2.3. Observation Indicators

Study investigators and data analysts remained blinded until all follow-up data were obtained, and the primary analytic strategies were finalized.

SAS and SDS were applied to evaluate the psychological state of patients in both groups before and after nursing. Mild anxiety refers to 59 points and below; moderate anxiety refers to 60–69 points; severe anxiety refers to 70 points and above; the higher the score, the more serious the anxiety. Mild depression refers to 53 points and below; moderate depression refers to 54–62 points; severe depression refers to 73 points and above; the higher the score, the more serious the depression.

KPS score: KPS score was used to assess the functional state. The higher the score, the better the health, the more tolerable the side effects of treatment on the body, and the higher adherence toward treatment. KPS score above 80 is interpreted as no need of external assistance to conduct daily life. A score of 50–70 is interpreted as need of partial external assistance to conduct daily life. A score below 50 is interpreted as total dependence on external assistance to conduct daily life.

ECOG score: ECOG was used to understand the general health and tolerance to treatment from the physical strength of the patient. Grade 0: the activity ability is completely normal, and there is no difference from the activity ability before the onset of the disease; grade 1: the tumor symptoms are mild, and the patient can walk freely and engage in light physical activities, including general housework or office work, but cannot engage in heavier physical activities; grade 2: the patient can tolerate the symptoms of the tumor, can walk freely and take care of himself, but has lost the ability to work, and the time spent in bed during the day does not exceed 50%; grade 3: the tumor symptoms are severe, the patient can only take care of himself partially, and the time spent in bed or wheelchair exceeds 50% during the day, but he can still get up and stand; grade 4: the disease is bedridden, and the patient cannot take care of himself; and grade 5: it denotes death.

QOL score: QOL score was applied to compare the QOL of patients in both groups. The full score is 100 points, and the lower the score, the worse the QOL of the patient.

Adverse reaction score: adverse reactions after chemotherapy include nausea, constipation, diarrhea, and hair loss. The total score is 10 points, and the higher the score, the more serious the adverse reaction.

### 2.4. Statistical Analysis

SPSS 20.0 was applied for data analysis software. Measurement data were represented as ($\bar{x}$ ± *s*), and the independent-samples *t*-test was applied for comparison. The counting data were represented as the number of cases (rate), and the chi-square test was applied for comparison. *P* < 0.05 was assumed as statistical significance. GraphPad Prism 8 was used for graphic rendering.

RETRACTED

## 3. Results

### 3.1. Comparison of the Baseline Data

In the control group, there were 27 men and 23 women; the age ranged from 28 to 64 years, with a mean age of 43.27 ± 15.34 years; among them, there were 8 cases of liver carcinoma, 10 cases of lung carcinoma, 9 cases of stomach carcinoma, 11 cases of breast carcinoma, 5 cases of colon carcinoma, and 7 cases of esophageal carcinoma. In the study group, there were 28 men and 22 women; the age ranged from 28 to 64 years, with a mean age of 43.36 ± 15.42 years; among them, there were 7 cases of liver carcinoma, 9 cases of lung carcinoma, 9 cases of stomach carcinoma, 12 cases of breast carcinoma, 7 cases of colon carcinoma, and 6 cases of esophageal carcinoma. There was no significant difference in baseline data such as gender, age, and cancer type between the control group and the study group (*P* > 0.05) (Table 1).

### 3.2. Comparison of SAS and SDS Scores

In the control group, the SAS scores of the patients before and after the intervention were 55.67 ± 8.46 and 49.68 ± 8.14, respectively; the SDS scores before and after intervention were 59.27 ± 6.48 and 55.47 ± 7.21, respectively. In the study group, the SAS scores of the patients before and after the intervention were 55.59 ± 8.48 and 42.17 ± 7.32, respectively; the SDS scores before and after intervention were 59.35 ± 6.51 and 49.22 ± 6.97, respectively. After nursing, the SAS and SDS scores of the study group were lower than those of the control group (*P* < 0.05) (Figure 1).

### 3.3. Comparison of KPS Score

The KPS scores of the patients in the control group before and after the intervention were 61.15 ± 7.12 and 68.31 ± 8.58, respectively; the KPS scores of the patients in the study group before and after the intervention were 61.20 ± 7.27 and 79.61 ± 10.22, respectively. After nursing, the KPS score of the study group was significantly higher than that of the control group (*P* < 0.05) (Figure 2).

### 3.4. Comparison of ECOG Score

The ECOG score of the patients in the control group before and after the intervention was 1.89 ± 0.27 and 1.61 ± 0.32; the ECOG score of the patients in the study group before and after the intervention was 1.88 ± 0.30 and 1.03 ± 0.25. After nursing intervention, the ECOG scores of the patients in the study group were significantly lower than those in the control group (*P* < 0.05) (Figure 3).

### 3.5. Comparison of QOL Score

The QOL score of the patients in the control group before and after the intervention was 57.21 ± 10.62 and 61.33 ± 10.35; the QOL score of the patients in the study group before and after the intervention was 57.18 ± 10.36 and 70.52 ± 12.39. After nursing intervention, the QOL score of the patients in the study group was significantly better than that of the patients in the control group (*P* < 0.05) (Figure 4).

RETRACTED

### 3.6. Comparison of Adverse Reaction Scores

Nausea, constipation, diarrhea, and hair loss scores of the control group were 8.91 ± 0.42, 7.63 ± 0.55, 7.55 ± 0.40, and 8.53 ± 0.72 and those of the study group were 7.16 ± 0.60, 6.17 ± 0.38, 5.72 ± 0.81, and 5.10 ± 1.14. The adverse reaction scores of the patients in the study group were lower than those in the control group (*P* < 0.05) (Table 2).

## 4. Discussion

Malignant tumor considerably threatens the human health and is regarded as a global health concern. The WHO survey shows that about 30% of cancer patients have missed the optimal treatment time at the time of diagnosis, and chemotherapy remains unavailable to alleviate the disease [9, 10]. At present, chemotherapy is the mainstay to prolong the life of patients with malignant tumors, but chemotherapy is associated with multiple side effects. As a result, patients are susceptible to psychological problems before chemotherapy, such as anxiety, fear, and depression, which requires good psychological care for patients before chemotherapy [11]. In this research, we compared the SAS and SDS scores of patients in both groups and found that there was no significant difference in the SAS and SDS scores of patients in both groups before the nursing intervention, but lower SAS and SDS scores of the patients in the study group after treatment, indicating that high-quality nursing intervention could help patients reduce the psychological pressure of the first chemotherapy for malignant tumors, reduce the psychological burden of the patients, and relieve the anxiety and fear of the patients. Psychological nursing is a part of high-quality nursing, and effective psychological nursing is an important means to enhance the QOL of patients with malignant tumors and promote the recovery of patients [12–15]. Most patients and their family members lack the corresponding knowledge of malignant tumor chemotherapy, and nurses should provide relevant disease treatment information to patients and their families in a timely manner during the whole process of chemotherapy. Applying high-quality nursing interventions and helping patients with targeted health education and guidance can allow patients to accept chemotherapy from both physical and psychological aspects, help patients reduce adverse reactions, and promote their physical recovery [16]. In this study, we compared the KPS, ECOG, and QOL scores of patients in both groups and found that the KPS, ECOG, and QOL scores of the patients in the study group were significantly higher than those in the control group after nursing intervention. The finding suggests that high-quality nursing intervention could effectively boost the patients' self-care ability, help the patients to enhance their tolerance to treatment, and thus improve the patients' QOL [17]. Additionally, adverse reactions in the early stage of chemotherapy, such as nausea, vomiting, constipation, diarrhea, hair loss, and other physical discomfort, can induce a greater psychological burden such as fear and resistance in patients and can also cause patients to experience negative world-weary emotions, leading to resistance to chemotherapy and hobbling the development of subsequent treatment [18, 19]. Consequently, there is an urgent need to comfort the patient, and high-quality nursing provides psychological comfort and psychological support in response to patients' adverse reactions. In this study, we found that the number of patients with adverse reactions of the study group was smaller than the control group patients, suggesting that high-quality nursing can effectively dredge patients' negative mood, give patients' spiritual support, and help patients face up to the follow-up treatment. This is presumably due to the fact that nursing staff could patiently explain the occurrence and prevention of adverse reactions to patients, so that patients are armed with a full understanding of adverse reactions and countermeasures, resulting in a sense of security physically and psychologically [20, 21].

RETRACTED

## 5. Conclusion

High-quality nursing intervention is a viable solution to reduce the psychological pressure of patients with malignant tumors with first chemotherapy, relieve patients' anxiety and fear, thus improve the chemotherapy effect, and enhance their QOL.

## Figures and Tables

**Figure 1:** Comparison of SAS and SDS scores. ^*∗∗∗*^*P* < 0.001.

**Figure 2:** Comparison of KPS scores. ^*∗∗∗*^*P* < 0.001.

**Figure 3:** Comparison of ECOG scores. ^*∗∗∗*^*P* < 0.001.

**Figure 4:** Comparison of QOL scores. ^*∗∗∗*^*P* < 0.001.

**Table 1:** Comparison of general data.

	Control group (*n* = 50)	Study group (*n* = 50)	*t* or *x*^2^	*P*
Gender (*n*)			0.04	0.841
Male	27	28		
Female	23	22		
Age ($\bar{x}$ ± *s*, years)	43.27 ± 15.34	43.36 ± 15.42	−0.029	0.977
Cancer type			0.573	0.989
Liver cancer	8	7		
Lung cancer	10	9		
Stomach cancer	9	9		
Breast cancer	11	12		
Bowel cancer	5	7		
Esophageal cancer	7	6		

**Table 2:** Comparison of adverse reaction scores ($\bar{x}$ ± *s*).

	Nausea	Constipation	Diarrhea	Hair loss
Control group (*n* = 50)	8.91 ± 0.42	7.63 ± 0.55	7.55 ± 0.40	8.53 ± 0.72
Study group (*n* = 50)	7.16 ± 0.60	6.17 ± 0.38	5.72 ± 0.81	5.10 ± 1.14
*t*	16.896	15.443	14.324	17.988
*P*	<0.01	<0.01	<0.01	<0.01

RETRACTED

## Data Availability

All data generated or analyzed during this study are included within the article.

## Abbreviation

QOL: Quality of life
SAS: Self-rating anxiety scale
SDS: Self-rating depression scale
KPS: Karnofsky performance status
ECOG: Eastern Cooperative Oncology Group
WHO: World Health Organization.
